# Evaluation of the Influence of Zhenwu Tang on the Pharmacokinetics of Digoxin in Rats Using HPLC-MS/MS

**DOI:** 10.1155/2021/2673183

**Published:** 2021-09-27

**Authors:** Chao Li, Dahu Liang, Yanhao Liu, Chaozhuang Shen, Xiaohu Wang, Bin Yang, Xianghong Li, Weijia Wang, Maodi Xu, Zhichen Pu, Hua Hu, Zijing Wu, Haitang Xie, Hua Sun

**Affiliations:** ^1^Yijishan Hospital of Wannan Medical College, No. 2, Zheshan West Road, Jinghu District, Wuhu 241000, China; ^2^Anhui Provincial Center for Drug Clinical Evaluation, Yijishan Hospital of Wannan Medical College, No. 2, Zheshan West Road, Jinghu District, Wuhu 241000, China; ^3^Department of Pharmacy, Bengbu First People's Hospital, No. 229, Tushan Road, Yuhui District, Bengbu 233000, China

## Abstract

Digoxin (DIG) is a positive inotropic drug with a narrow therapeutic window that is used in the clinic for heart failure. The active efflux transporter of DIG, P-glycoprotein (P-gp), mediates DIG absorption and excretion in rats and humans. Up to date, several studies have shown that the ginger and Poria extracts in Zhenwu Tang (ZWT) affect P-gp transport activity. This study aimed to explore the effects of ZWT on the tissue distribution and pharmacokinetics of DIG in rats. The deionized water or ZWT (18.75 g/kg) was orally administered to male Sprague–Dawley rats once a day for 14 days as a pretreatment. On day 15, 1 hour after receiving deionized water or ZWT, the rats were given the solution of DIG at 0.045 mg/kg dose, and the collection of blood samples was carried out from the fundus vein or excised tissues at various time points. HPLC-MS/MS was used for the determination of the DIG concentrations in the plasma and the tissues under investigation. The pharmacokinetic interactions between DIG and ZWT after oral coadministration in rats revealed significant reductions in DIG C_max_ and AUC_0-∞_, as well as significant increases in T_1/2_ and MRT_0-∞_. When coadministered with ZWT, the DIG concentration in four of the investigated tissues statistically decreased at different time points except for the stomach. This study found that combining DIG with ZWT reduced not only DIG plasma exposure but also DIG accumulation in tissues (heart, liver, lungs, and kidneys). The findings of our study could help to improve the drug's validity and safety in clinical applications and provide a pharmacological basis for the combined use of DIG and ZWT.

## 1. Introduction

Zhenwu Tang, also known as Xuanwu tang, is a representative prescription for warming yang and promoting urination in “Treatise on febrile diseases”, consisting of Poria, Radix Paeoniae Alba, Aconiti Lateralis Radix Praeparata, Rhizoma Atractylodis macrocephalae, and ginger [1, 2]. This formulation has been widely used in the last decades, and as modern researchers continue to research Zhenwu decoction in detail, its clinical use is expanding to include cardiovascular, urinary, neurological, and other system diseases [3, 4]. DIG is one of the most well-known medications in cardiovascular medicine, but it has a narrow therapeutic window [5–7]. The US Food and Drug Administration (FDA) has approved it for the effective management and treatment of heart failure, and it received an IIb-B recommendation in the European Society of Cardiology's 2016 heart failure guidelines [8].

DIG is the substrate of P-glycoprotein (P-gp, active efflux transporter) and is often used as the probe drug for P-gp [9]. Furthermore, P-gp is widely distributed in the tissues of humans and rats, especially in the basal parietal surface of intestinal epithelial cells, bile tubules, and proximal renal tubules [10–12]. He et al. and Kim et al. have already disclosed that the extracts of ginger and Poria in Zhenwu Tang affect the transport function of P-gp [13, 14].

According to the recommendations for rational use of drugs for heart failure in China (2019), combining traditional Chinese medicine and western medicine will not only improve the curative effect but also reduce the side effects [15]. DIG is the representative medicine of digitalis listed in the guideline, and Zhenwu Tang is also one of the traditional Chinese medicines used as adjuvant therapy for the treatment of heart failure listed in the guideline [15]. Clinical studies have shown that the DIG, when used in combination with ZWT for treating heart failure, has shown to be more effective than either drug alone [16, 17]. As mentioned above, patients who receive DIG may have a simultaneous intake of ZWT, and this may affect the pharmacokinetic properties of DIG. However, information about the interaction between DIG and ZWT is lacking. Therefore, this research aimed to see how ZWT affected DIG tissue distribution and pharmacokinetics.

## 2. Materials and Methods

### 2.1. Preparation of Zhenwu Tang

Raw materials of *Rhizoma Atractylodis macrocephalae, Poria, ginger, Radix Paeoniae Alba,* and *Aconiti Lateralis Radix Praeparata*, which were provided by the Yijishan Hospital of Wannan Medical College (Wuhu, China), were crushed into powder in a weight ratio of 2 : 3 : 3 : 3 : 1 [18]. This was followed by the maceration of the mixture in water (10 : 1, v/w) for half an hour before being decocted for 1.5 h. The mixture was filtered with a vacuum filtration device supplied by Qingdao SuYuan environmental protection equipment Co., Ltd (Qingdao, China). After filtration, the decoction was collected, and the residual was decocted for 0.5 h with water (1 : 8, w/v). Two parts of decocted solutions were pooled and concentrated utilizing rotary evaporators at about 80°C, and then, the concentrated extract was dried and pulverized to obtain the ZWT extract powder at a yield of 15.92% (w/w, dried powder/crude herbs). The drying oven for drying was provided by Jiangsu Spring Instrument Co., Ltd (Jiangsu, China), and the pulverizer supplied by Shanghai SiJun Machinery Equipment Co., Ltd (Shanghai, China) was utilized to crush raw materials and the dried extract.

Following preparation, the dried powder was stored at room temperature for further use.

### 2.2. Materials and Reagents

The reference standard of DIG (batch No: 20181221) with a purity of >98% was obtained from Hefei Ruijie Bio-Technology Co., Ltd. Lappaconitine hydrobromide with a purity of >98% was provided by the Shanghai Yuanye Bio-Technology Co., Ltd. (Shanghai, China) and was used as internal standard (IS). HPLC-grade formic acid and methanol were provided by Merck (Darmstadt, Germany). Similarly, ethyl acetate and acetonitrile were of HPLC grade and were obtained from Tedia, Fairfield, USA. Water was prepared with a Milli-Q system (Millipore, USA) for this study. All other reagents used were of analytical grade.

### 2.3. Animals

Fifty-six healthy male Sprague–Dawley rats (at 5 weeks old), weighing 180–220 g, were supplied by Shushan Animal Breeding Farm (Hefei, China). All animals were fed on standard chow in a climate-controlled facility at 22 ± 2°C and relative humidity 50 ± 10% with dark/light cycle of 12 h and were given free access to water ad libitum. The standard chow was purchased from Beijing Fubo Biological Technology Co., Ltd (Beijing, China). All animals were housed in IVC cages (420*∗*250*∗*230 MM) and fasted for 24 h but provided with plenty of water before initiation of the experiment. In order to prevent contamination, the rats were housed in an intelligent IVC system and the corn cob bedding (6 mesh) in the cages was changed daily. All of this study's protocols and welfare on animals were approved by the Animal Ethics Committee of Wannan Medical College (March 8, 2021; No: 2021-074).

### 2.4. Pharmacokinetic Study

For pharmacokinetic studies, sixteen male SD rats were randomly divided into two groups (*n* = 8): (1) DIG alone and (2) DIG + ZWT. DIG and ZWT were dissolved in deionized, water and the solutions were administered via gavage. The dosage of ZWT for SD rats was kept as 18.75 g/kg based on the previously reported study. The rats in the DIG alone group were given 2 mL of deionized water once a day for 14 days as a pretreatment. For the DIG + ZWT group, the rats were pretreated with ZWT at a dose of 18.75 g/kg (equivalent to 2.99 g·kg^−1^ZWT extract powder) for 14 days. On day 15, 1 hour after receiving deionized water or ZWT, the rats in both groups were given the solution of DIG at 0.045 mg/kg dose. The collection of serial blood samples (approximately 450 *μ*L) was carried out from the fundus vein into heparinized tubes at various intervals (0, 0.17, 0.33, 0.5, 0.75, 1, 1.5, 2, 3, 4, 6, 8, and 12 h) after DIG administration. The plasma was obtained by centrifuging the blood samples for 10 min at 4000 rpm. Plasma samples were then frozen at −80°C until bioanalysis.

### 2.5. Tissue Distribution Study

For investigating the effect of ZWT on the tissue distribution of DIG in rat main tissues, forty male SD rats were randomly divided into two groups as mentioned in the previous section. The dose and period of administration for each group were the same as those described in the pharmacokinetic study section. Before the rats were sacrificed, blood samples were obtained from the fundus vein into heparinized tubes and then were subjected to centrifugation for 5 min at 4000 rpm to obtain plasma. Then, the rats were sacrificed by cervical dislocation at 0.5 h, 1h, 2 h, 4 h, and 8 h after taking DIG orally (four animals per time point), respectively. The heart, liver, lungs, kidneys, and stomach tissues were immediately excised, rinsed thoroughly with ice-cold phosphate-buffered saline (PBS), dried with filter paper, and stored at −80°C. The tissue samples were ground with precooling phosphate-buffered saline (PBS) at a ratio of 3 : 1 (v/w) to prepare tissue homogenate for use during the study. The digoxin concentrations in the investigated tissues were indicated in ng/g while using the formula C_T_ = C_S_ × V_S_/W_S_, in which CT indicates the tissue concentration (ng/g), and Vs and C_S_ are the volume (mL) and concentration (ng/mL) of the tissue homogenate, while W_S_ represents the weight (g) of tissue samples, respectively.

### 2.6. Sample Preparation

The working solution of IS (20 *μ*L, 500 ng/mL) was mixed with plasma samples (200 *μ*L), vortex-mixed for 5 minutes, and then extracted with 1 ml ethyl acetate. After shaking for 10 min, the mixture was subjected to centrifugation at 4000 rpm for 10 min at 4°C. This was followed by moving the supernatant to a new centrifuge tube and dried under nitrogen at 45°C before being redissolved in a 70% acetonitrile-water mixture (100 *μ*L). The solution was then shaken for 5 min before being subjected to centrifugation for 10 min at 12000 rpm. The supernatant was transferred to an autosampler vial, and 15 *μ*L of the supernatant was injected into the HPLC-MS/MS system. Small tissue slices were individually weighed and homogenized with a 3-fold volume of ice-cold phosphate-buffered saline (PBS). A 50 *μ*L IS (250 ng/ml) was aliquoted in a centrifuge tube and then spiked with 500 *μ*L homogenate followed by the addition of 2.5 mL ethyl acetate to extract. The mixture was treated in the same way as the plasma treatment described above. The supernatant was then subjected to an HPLC-MS/MS analysis.

### 2.7. HPLC-MS/MS Instrument and Conditions

For HPLC, CTO-10ASvp column oven, SIL-HTc autosampler (Shimadzu, Japan), and Shimadzu LC-20AD binary pump were used in the study. An Agilent ZORBAX Eclipse XDB-C18 (5 *μ*m, 4.6 × 150 mm) column was used for accomplishing the chromatographic separation with the mobile phase consisting of 70% acetonitrile-water (comprising 10 mmol ammonium acetate and 0.1% formic acid) at a flow rate of 0.5 mL/min. The injection volume was 15 *μ*L, and the column temperature was held at 30°C.

In a positive ion mode, an API 4000 triple quadrupole tandem mass spectrometer with an ESI source was used, and the acquisition and analysis of data were done with Analyst 1.6.2 software (Applied Biosystems Sciex, USA). Multiple reaction monitoring (MRM) parameters for the DIG and lappaconitine hydrobromide (IS) were optimized and are summarized in Table 1. The other parameters for ionization were as follows: curtain gas, 20 psi; collision gas, 6 psi; ion source gas 1, 50 psi; ion source gas 2, 50 psi, respectively, with a temperature of 500°C and an ion spray needle voltage of 5500 V.

### 2.8. Method Validation

The bioanalytical method validation guidance for industry released by the FDA in 2018 was used to validate the analytical approach used in this study [19]. The selectivity, specificity, precision, linearity, accuracy, matrix effects, stability, and recovery were used as key metrics to affirm the validity of this method.

#### 2.8.1. Specificity and Selectivity

Tissue and plasma homogenates from six individual rats were tested for specificity and selectivity to assess possible interferences at the LC peak region for IS and analytes. The chromatograms of tissue homogenates (liver was chosen as the representative tissue) and blank plasma were compared to those of tissue homogenates and normal plasma spiked with analytes and IS, as well as homologous samples after an oral dose.

#### 2.8.2. Determination of Linearity and Lower Limits of Quantification (LLOQ)

The calibration curve was generated by plotting the ratio of peak areas of DIG and lappaconitine hydrobromide against the DIG standard concentrations of plasma and tissue homogenate by the least-square method using 1/*x*^2^ as the weighting factor. The content of DIG in the test samples was calculated using the obtained standard curve. The determination of the analytes' LLOQ was carried out at the lowest detectable concentration while taking into account a 10 : 1 noise-calibration baseline point ratio, which can be quantified with accuracy and precision being less than 20%, evaluated by samples analysis in six replicate analyses.

#### 2.8.3. Accuracy and Precision

The accuracy and intraday precision were investigated by evaluating the QC samples of plasma and tissue homogenate (liver was chosen as the representative tissue) at high, medium, and low concentrations using six replicates during the same day. The accuracy and interday precision were measured via analyzing the same replicate samples on three consecutive days. The accuracy of the analytical approach used in this study was investigated by calculating the measured analyte concentration to its nominal value and was expressed as the relative error (RE). The precision was expressed as relative standard deviation (RSD).

#### 2.8.4. Recovery and Matrix Effect

The extraction recovery rate of the analyte was assessed by analyzing six replicates of QC plasma or tissue homogenate samples, with the liver being the representative tissue, at high, medium, and low concentrations. It was determined by comparing the response of QC samples spiked with the analyte before extraction to the response of samples spiked at homologous concentrations after extraction. The effect of the matrix was evaluated similarly. The effects of the matrix were calculated by comparing the response obtained from samples where the extracted matrix (blank plasma and tissue homogenate) was spiked with quality control solution with those obtained by adding the same concentration of analyte in 50% methanol in water.

#### 2.8.5. Stability

DIG stability in tissue homogenate samples and plasma was assessed by examining QC samples that had been stored under various conditions for various periods. QC samples were exposed at room temperature for 4 h before preparation to assess pretreatment stability, while autosampler stability was tested by storing samples in the autosampler for 24 h. The long-term stability of QC samples was tested by storing them at −80°C for 15 days. QC samples were regularly frozen and thawed for three cycles from −80°C to 25°C for freeze-thaw period stability testing.

### 2.9. Statistical Analysis

The mean ± standard error was used to display all of the results. The pharmacokinetic parameters were calculated using noncompartmental model via the Phoenix WinNonlin software (v8.1, CERTARA, NJ, USA) except the C_max_ and T_max_ which were directly acquired from the experimental data. For the study of tissue distribution, the DIG contents of rat tissue samples were presented in the form of ng/g. *T*-tests were employed for the comparison between the data of two independent groups and accomplished by SPSS 25.0 software (SPSS, Inc., IL, USA). When *P* < 0.05, the differences were considered to be significant.

## 3. Results

### 3.1. Optimization of HPLC-MS/MS Conditions

Some mobile phases, such as methanol-water and acetonitrile-water, were investigated for achieving optimized chromatographic behavior. Finally, the acetonitrile-water system was found to enhance the sensitivity of this method. Furthermore, after researching a series of buffers and acid-base solutions in combination with the acetonitrile-water system, the addition of formic acid (0.1%) to the water phase could improve the signal response of DIG and lappaconitine hydrobromide remarkably, while the ammonium acetate would improve their peak shape. Therefore, the mobile phase containing 70% acetonitrile and 30% water (0.1% formic acid, 10 mmol ammonium acetate) was utilized in this method. With a flow rate of 0.5 mL/min, the column temperature was held at 30°C.

The signal-to-noise ratio in positive and negative ion modes was tested in our study, and we found the positive ion mode would produce a better signal-to-noise ratio.  Figure 1 illustrates the MS/MS product ion spectra of the DIG and lappaconitine hydrobromide. The optimized MS parameters such as declustering potential and collision energy were researched to enhance the sensitivity, and the optimized values are all summarized in Table 1. This combination resulted in reduced background noise, improved peak shape, shorter running times, and improved DIG and IS response.

### 3.2. Method Validation

#### 3.2.1. Specificity and Selectivity

The analytical method's specificity and selectivity for DIG and IS were investigated by comparing blank plasma chromatograms with the corresponding spiked plasma and blank rat tissue homogenate with the corresponding spiked rat tissue homogenate in LLOQ.  Figure 2 shows representative MRM chromatograms. At the retention times of SI and DIG, no major interferences of endogenous substances in rat plasma and tissue homogenate were identified, and the method demonstrated good specificity.

#### 3.2.2. Linearity and LLOQ

The correlation coefficients, regression equations, and the linear ranges of DIG are summarized in Table 2. The LLOQ of DIG was 0.05 ng/mL in heart, plasma, lung, and kidney samples, while it was 0.1 ng/ml in liver and stomach samples. These regression equations were sufficient to facilitate tissue distribution studies and pharmacokinetic analyses.

#### 3.2.3. Precision and Accuracy

Table 3 summarizes the accuracy and precision data of the analytical method used in this study. The interday and intraday precision (RSD) and accuracy (RE) of QC samples of tissue homogenates and plasma were consistent with the study's acceptance criteria.

#### 3.2.4. Matrix Effect and Extraction Recovery

Table 4 shows the matrix effects and DIG extraction recovery. The extraction recovery of DIG from spiked rat plasma and tissue homogenate samples was all over 68% in different samples at high, medium, and low concentrations. The matrix effect of DIG was in the range of 101.33–103.12% for plasma and 102.54–108.89 for tissue samples (with the liver being chosen as representative tissue), thus indicating that there was no major matrix impact for the DIG.

#### 3.2.5. Stability

Table 5 summarizes the stability of tissue homogenate and DIG in plasma over a variety of temperature and time conditions. The results of a series of stability were all within the acceptable limit, suggesting that the DIG is stable in plasma and tissue homogenate under preparation and storage conditions.

### 3.3. Effect of Zhenwu Tang on Pharmacokinetics of Digoixn in Rats

Figure 3 depicts the mean plasma concentration of DIG vs. time profiles, and Table 6 outlines the pharmacokinetic changes of DIG. Upon coadministration with 18.75 g/kg of ZWT, the AUC_0-∞_ and AUC_0-t_ of DIG both decreased by almost 50%. Also, the values of MRT_0-∞_ of digoxin were delayed from 4.02 h in the DIG alone group to 5.08 h (*P* < 0.05) after coadministration of DIG with ZWT. Furthermore, after DIG cotreatment with ZWT, the T_1/2_ of DIG was significantly increased when compared to the DIG alone group. However, in the DIG alone group, the mean C_max_ of DIG was 1.4-fold of that of the DIG + ZWT group. The CL of DIG tended to be increased from 4.42 to 7.85 L/h/kg, whereas no statistically significant difference was found between the DIG alone group and the cotreatment group.

### 3.4. Zhenwu Tang Effects on the Tissue Distribution of Digoxin in Rats

The DIG concentrations in rat's five major tissues including heart, liver, lung, kidneys, and stomach and plasma were investigated. As illustrated in Figure 4, when coadministered with ZWT, the DIG concentration in four of the investigated tissues statistically decreased at different time points (*P* < 0.05) except the stomach, in which the DIG concentration lacked statistical differences between the DIG alone group and cotreatment group (*P* > 0.05). In comparison with other tissues, the concentration of DIG was found the highest in the liver of the rats in both cases of DIG alone or DIG + ZWT group at each time point except in 0.5 h. At 0.5, 1, and 4 h after treatment, plasma concentrations of DIG in the DIG + ZWT group were reduced to 22, 66, and 22% of those in the DIG alone group, respectively.

## 4. Discussion

We developed and validated a sensitive and rapid HPLC-MS/MS method for measuring DIG concentrations in plasma and tissues, which was subsequently used in this research. For the first time, our study investigates the influence of ZWT on DIG absorption and distribution. Furthermore, DIG exposure in plasma and primary organs offers basic knowledge for treatment outcomes of DIG and ZWT combination treatment.

Since DIG is the substrate of P-gp, and if coadministered with P-gp inducers or inhibitors, it may affect the pharmacokinetic properties of DIG. In our study, the pharmacokinetics of DIG in rats after oral administration of DIG with and without ZWT were investigated. Previous studies have reported that the DIG with a narrow therapeutic window would lead to a range of adverse reactions ranging from vomiting, nausea, visual impairment to ventricular fibrillation, and even eventual death [20–22]. Our study found that combining DIG with ZWT not only decreased plasma exposure to DIG but also decreased DIG accumulation in tissues (heart, liver, lung, and kidney), which would help reduce the incidence of adverse events. These findings may have far-reaching clinical implications. The drug-drug interaction (DDI) is usually detected in the clinic by measuring drug plasma concentrations [23]. Nevertheless, the DDI mediated by specific transporter might exist even if there is no significant statistical change in blood concentration [24, 25]. The concentrations of DIG in the plasma and investigated tissues of the DIG + ZWT group appeared to be lower at certain designed time points of this study relative to the DIG alone group, despite no statistically significant difference being observed. This phenomenon may be due to the small number of experimental cases used in this research.

Theoretically, inhibiting or enhancing the function of P-gp may affect its substrate plasma exposure in rats and humans [26, 27]. Previous studies indicated that the DIG is the substrate of P-gp and is frequently used as the probe drug for P-gp [28–30]. Chung et al. have already disclosed that the six kaempferol derivatives extracted from ginger in ZWT have shown a P-gp regulation effect [31]. In addition, Li et al. have demonstrated that triterpenoids from Poria could effectively regulate the activity of P-gp in many MDR cell lines [32]. These findings suggest that the induction of P-gp of the components in ZWT may be responsible for the decrease in digoxin accumulation in plasma and organs observed in this research.

The heart, spleen, liver, lung, kidney, stomach, and testis were all collected for this tissue distribution study. While DIG concentrations in the spleen and testis of rats in the DIG alone group could be detected, DIG concentrations in the spleen and testis of rats in the DIG + ZWT group were lower than our developed method's lower limit of quantification. Therefore, in this report, we only enumerated and compared the DIG concentration in the liver, heart, kidney, lung, and stomach instead of spleen and testis.

Studies have already shown that the combination of ginger and Aconiti Lateralis Radix Praeparata in ZWT could enhance myocardial contractility, reduce myocardial oxygen consumption, alleviate arrhythmias, and thus produce the effect of anti-heart failure [33–35]. Ye et al. have already disclosed that the combined use of DIG and ZWT for treating heart failure has shown to be more effective than DIG alone [17]. In summary, when DIG is used in combination with ZWT, the blood concentration of DIG decreased, but the therapeutic effect on heart failure increased, which might be due to the synergistic anti-cardiac failure effect of DIG and ZWT.

At present, we have only evaluated the effects of ZWT on the tissue distribution and pharmacokinetics of DIG in rats when the two drugs were used together but have not studied whether the latter would have any impact on the former. Therefore, in subsequent experiments, we will conduct a supplementary study. Finally, the drawbacks and benefits of combining DIG and ZWT will be investigated further.

## 5. Conclusion

The effects of Zhenwu Tang on digoxin tissue distribution and pharmacokinetics were investigated in this research. The results showed that the tissue distribution and pharmacokinetic profiles of digoxin were altered after Zhenwu Tang oral administration in rats. Coadministration with Zhenwu Tang (18.75 g/kg) reduced not only digoxin plasma exposure but also digoxin accumulation in tissues (heart, liver, lungs, and kidneys).

## Figures and Tables

**Figure 1:** Mass spectrum of multireaction monitoring of digoxin (a) and the lappaconitine hydrobromide (IS) (b).

**Figure 2:** Representative chromatograms of blank rat plasma (a) and liver homogenate (b); blank rat plasma (c) and liver homogenate (d) spiked with digoxin in LLOQ and lappaconitine hydrobromide; plasma sample (e) at 1h after an oral administration of pure digoxin and liver homogenate (f) after an oral administration of pure digoxin. (A) represents digoxin, and (B) represents IS.

**Figure 3:** The mean plasma concentration of digoxin vs. time profiles after digoxin oral administration in rats at 0.045 mg/kg dose in the absence and presence of ZWT (18.75 g/kg) (*n* = 8).

**Figure 4:** Tissue distribution of digoxin in rat plasma, heart, liver, lung, kidney, and stomach samples (*n* = 4).

**Table 1:** Optimized MRM parameters for analytes and IS.

Analyte	Molecular formula	Precursor ion (*m*/*z*)	Product ion (*m*/*z*)	Declustering potential	Collision energy
Digoxin	C_41_H_64_O_14_	798.7	651.5	65	17
Lappaconitine hydrobromide	C_32_H_45_BrN_2_O_8_	585.3	162.0	110	57

**Table 2:** Summary of the correlation coefficients, linear regression equation, and the linear ranges of digoxin in rat plasma and tissue homogenate samples.

Sample	Regression equation	*R* ^2^	Linear range (ng/mL)
Plasma	*y* = 0.00065*x* + 0.0429	0.9946	0.05–10
Heart	*y* = 0.00125*x* + 0.0470	0.9928	0.05–10
Liver	*y* = 0.00079*x* + 0.0001	0.9974	0.1–20
Lung	*y* = 0.00124*x* + 0.0470	0.9936	0.05–10
Kidney	*y* = 0.00804*x* + 0.0596	0.9978	0.05–10
Stomach	*y* = 0.00284*x* + 0.0004	0.9958	0.1–20

**Table 3:** The accuracy and precision for digoxin in rat plasma and liver homogenate (6 replicate samples per concentration).

Biosamples	Spiked conc (ng/mL)	Intraday (*n* = 6)			Interday (*n* = 6 × 3)		
		Measured conc (ng/ml)	Precision (RSD, %)	Accuracy (RE, %)	Measured conc (ng/ml)	Precision (RSD, %)	Accuracy (RE, %)
Plasma	0.05	0.05 **±** 0.00	4.46	0.05	0.05 **±** 0.00	5.56	2.05
	0.15	0.14 **±** 0.02	12.35	0.82	0.15 **±** 0.02	10.45	0.18
	1.2	1.23 **±** 0.13	10.20	−0.31	1.27 **±** 0.12	9.82	5.75
	8	8.80 **±** 0.41	4.70	11.83	8.87 **±** 0.26	2.88	10.87

Liver	0.1	0.10 **±** 0.01	10.07	−4.98	0.09 **±** 0.01	7.63	−8.58
	0.3	0.28 **±** 0.02	8.52	−7.61	0.28 **±** 0.02	6.93	−5.55
	2	1.79 **±** 0.14	8.09	−10.44	1.85 **±** 0.15	7.80	−7.86
	16	16.69 **±** 1.37	8.21	4.34	16.26 **±** 1.25	7.70	3.84

**Table 4:** The matrix effects and extraction recovery of digoxin in liver homogenate and rat plasma (*n* = 6).

Biosamples	Conc. (ng/mL)	Extraction recovery (mean ± SD)	Matric effect (mean ± SD)
Plasma	0.15	76.02 **±** 7.61	101.33 **±** 8.37
	1.2	75.04 **±** 7.66	101.81 **±** 13.62
	8	71.25 **±** 4.41	103.12 **±** 14.74

Liver	0.3	68.45 **±** 3.00	108.89 ± 12.25
	2	74.74 **±** 5.41	103.68 **±** 7.54
	16	75.33 **±** 5.87	102.54 **±** 11.20

**Table 5:** Stability of digoxin in plasma and liver homogenate biosamples under a variety of conditions (*n* = 6).

Sample	Spiked conc. (ng/mL)	Pretreatment stability (at room temperature for 4 h)			Autosampler stability (at room temperature for 24 h)			Long-term stability (at −80°C for 15 days)			Freeze-thaw cycle stability (at −80°C)		
		Concentration found		RSD (%)	Concentration found		RSD (%)	Concentration found		RSD (%)	Concentration found		RSD (%)
		Mean	SD		Mean	SD		Mean	SD		Mean	SD	
Plasma	0.15	0.17	0.01	3.91	0.16	0.01	7.40	0.14	0.01	8.07	0.14	0.01	6.38
	8	9.09	0.20	2.19	8.99	0.14	1.61	8.58	0.31	3.65	8.80	0.54	6.14

Liver	0.3	0.30	0.03	10.54	0.32	0.02	5.75	0.28	0.02	6.58	0.30	0.03	11.60
	16	17.62	0.90	5.12	16.82	1.47	8.76	16.30	1.37	8.38	16.21	1.90	11.71

**Table 6:** Digoxin oral pharmacokinetic parameters after oral administration in rats at 0.045 mg/kg dose alone or together with ZWT (18.75 g/kg) (*n* = 8).

Group	T_1/2_ (h)	*T*_max_ (h)	MRT_0-∞_ (h)	*C*_max_ (ng·mL^−1^)	CL/F (L/h/kg)	AUC_0-t_ (ng·mL^−1^·h)	AUC_0-∞_ (ng·mL^−1^·h)
DIG	2.75 ± 0.18	0.41 ± 0.11	4.02 ± 0.24	3.29 ± 0.49	4.42 ± 0.70	10.48 ± 1.78	12.27 ± 1.94
DIG + ZWT	3.47 ± 0.75^*∗∗*^	0.60 ± 0.15	5.08 ± 0.86^*∗*^	2.35 ± 0.23^*∗*^	7.85 ± 0.83	5.18 ± 0.59^*∗∗*^	6.13 ± 0.55^*∗∗*^

^*∗*^*P* < 0.05, ^*∗∗*^*P* < 0.01 vs. DIG alone group.

## Data Availability

The data that support the findings of this study are available on request from the corresponding author. The data are not publicly available due to their containing information that could compromise the privacy of the researcher.
